# Expression of SR-BI and LXR*α* in Macrophage Origin Foam Cells of Mouse RAW264.7 Up-regulated by Astragalus Polysaccharide

**DOI:** 10.1155/2022/3920584

**Published:** 2022-09-27

**Authors:** Lichen Yan, Jing Guo, Xiaohua Gao

**Affiliations:** ^1^Department of Gastroenterology, Jincheng People's Hospital of Shanxi, Jincheng 048000, Shanxi, China; ^2^Heping Hospital Affiliated to Changzhi Medical College, Changzhi 046000, Shanxi, China

## Abstract

**Objective:**

To investigate the influences of *Astragalus* polysaccharides (APS) on the expressions of SR-BI(Scavenger receptor-BI) and LXR *α* in RAW264.7 macrophage origin foam cells.

**Methods:**

Mouse RAW264.7 cells were induced in foam cells and identification of the foamed by oil-red O staining. The RAW264.7 macrophage origin foam cells were dealt with APS with distinct contents (0, 10, 20, 50, or 100 mg/L). The mRNA and protein expressions of SR-BI and LXR*α* were measured by RT-PCR as well as ELISA, respectively.

**Results:**

Macrophages were differentiated into foam cells 48 h after ox-LDL induction. In contrast to the control part, the mRNA and protein expressions of SR-BI and LXR*α* in RAW264.7 macrophage origin foam cells were up-regulated dosage-dependently after being treated with different concentrations of APS (*P* < 0.05).

**Conclusion:**

APS could promote intracellular cholesterol efflux by up-regulating the expressions of SR-BI and LXR *α* of RAW264.7 cells.

## 1. Introduction

Atherosclerosis (AS) is the primary pathological foundation of cardiovascular diseases, which is a serious threat to human health. AS injury has characteristics of cholesterol deposition because of cholesterol metabolism imbalance. The dysfunction of cholesterol metabolism in macrophages is an important mechanism of AS. Therefore, how to reduce cholesterol intake and promote cholesterol efflux is the key to prevent AS. Macrophages have unlimited uptake of oxidized modified cholesterol, so cholesterol efflux plays an important role in inhibiting its blistering [1] and is regulated by related transporters and receptors. Studies have indicated that Scavenger receptor I (SR-BI) can make cholesterol flow from cells to HDL particles, mediate the binding of HDL to cholesterol, and thereby esterify cholesterol into cholesterol ester [2, 3]. Hepatic X receptor *α* (LXR*α*) can transport excess cholesterol to the liver for transformation and clearance through plasma HDL [4]. *Astragalus* polysaccharides (APS), an active ingredient extracted from *Astragalus* membranaceus, is vital for lipid modulation and AS prevention. Its main biological activities include antioxidation, immunity enhancement, antitumor, blood glucose regulation, antiatherosclerosis and other functions. Previous studies have found that it had a significant effect on lipid regulation and prevention of AS. In in vitro experiments, it had been confirmed that APS could enhance the phagocytic activity of macrophages that acted on low-density lipoprotein, enhance the ability to clear pathological lipids, and APS had a certain inhibition effect on the accumulation of lipids in macrophages.

In this study, RAW264.7 macrophages were considered as study objects to observe effects of APS on expression of SR-BI, LXR*α* mRNA, and protein, and then explore the possible mechanism of APS on cholesterol reverse transport.

## 2. Materials and Methods

### 2.1. Materials

RAW264.7 murine macrophages strain (Cell Bank, Shanghai Institution of Cellular Biology, CAS); *Astragalus* polysaccharides (APS) (Xi'an Watson Biotechnology Co., Ltd.); DMEM cultivation intermediary, FBS and trypsin (Hyclone); low-density lipoprotein (LDL) (Shanghai Shenggong Bioengineering Co., LTD.); total RNA extraction kit (Bomide Biotechnology Co., Ltd.); RT-PCR kit (Nanjing KGI Biology Co., Ltd.); *β*-actin, SR-Bi and LXR*α* were synthesized by Shanghai Sangon. ELISA kit (Shanghai Chaoyan Biotechnology Co., Ltd.) and other reagents are imported or domestic analytical reagents.

### 2.2. Treatment of Dialysis Membrane

Small segments of 20–30 cm were cut from the intact dialysis membrane, and the dialysis membrane was moistened and boiled in 10 mmol/L NaHCO_3_ solution for 10 min, and then boiled in 10 mmol/L EDTA for 10 min, and repeated once. After it was cleaned with distilled water, it was put in 20%–50% ethanol solution and was stored at 4°C. It was ensured that the dialysis bag was always infiltrated in the ethanol solution to prevent the growth of cellulolytic microorganisms.

### 2.3. Oxidative Modification and Identification of Low-Density Lipoprotein

PBS (0.01 mol/L, pH 7.2) was used to adjust LDL concentration to 1.6 g/L, and CuSO_4_ was added to make the final concentration of LDL solution to 10 *μ*mol/L. The solution was fully oxidized at 37°C for 20 h, and then put into a dialysis bag. The oxidation was terminated with PBS solution containing 100 *μ*mol/L ethylenediamine tetra acetic acid at 4°C for 24 h. Low-density lipoprotein was filtered by a 0.45 *μ*m membrane, and then protein quantification used BCA reagent. Regulatory protein concentration was 1 g/L as well as kept under 4°C for later utilization.

### 2.4. Cell Cultivation and Experimental Grouping

RAW264.7 cells could be cultivated with DMEM including 10% FBS under the condition of 37°C and 5% CO_2_, and 1.0 × 10^5^ U/L penicillin as well as 1.0 × 10^5^ U/L streptomycin were supplemented into the cultivation medium, respectively. When the cells entered the logarithmic growth phase, they were treated experimentally. The cells could be cultivated in a medium including 50 mg/L ox-LDL for 48 h to induce them to become foam cells. Oil red O dyeing could be applied to observe solution deposition in the cells, and then the cells were separated in random parts for the experiment. No disposal was conducted on the control part, and the experimental part was incubated with APS with concentration of 10, 20, 50, and 100 mg/L for 24 h, respectively.

### 2.5. Oil Red O Staining

RAW264.7 cells were cultivated in a 6-hole cultivation dish using disinfection with glass. 48 h after ox-LDL differentiation was induced, PBS solution was washed 3 times, 50% isopropyl alcohol was fixed for 1 min, and then absorbed with fixative solution, and colored with red O staining liquid at room temperature for 10 min. Hematoxylin was dyed for 5 minutes. The tablets were sealed with hydrochloric acid and ethanol for blue staining and microscope observation.

### 2.6. mRNA Expression of SR-BI and LXR*α* Detected via RT-PCR

Various groups of cells were collected. Total RNA was drawn based on illustrations of the Trizol kit, and the RNA could be reversely transcribed to cDNA based on illustrations, and reverse transcription products were taken for PCR. After predenaturation under 94°C for five minutes and PCR amplification for 33 cycles (denaturation under 94°C for thirty seconds, annealing for 45 s, extension under 72°C for one minute), they were extended at 72°C for 10 min.

The primers were synthesized by Shanghai Sangon, SR-BI: upstream: 5′-TGAAGGAAGGAAGAGCCTAAGA-3′, downstream: 5′-CACACACACACACACACACAAA-3′, the amplified fragment length was 223 bp; LXR*α*: upstream: 5′-CTCCAGCCCCTCTCTCTTTATT-3′, downstream: 5′-GGATTTCTTTCAGCAAC.

CATCT-3′, the amplified fragment length was 214 bp; *β*-actin was selected as the inner control, and the primer sequence was below: upstream: 5′-ATATCGCTGCGCTGGTCGTC-3′, downstream: 5′-AGGATGGCGTGAGGGAGA.

GC-3′, the amplified fragment length was 517 bp. The extracted RNA was amplified in different PCR tubes with the same conditions, and after the reaction ended, 10 *μ*L of reaction products were taken to carry out 2.5% AGE as well as ethidium bromide dyeing. Then, a picture of gel image analysis system was taken, the light absorption values of target genes and internal genes in each group were analyzed, and the ratio of the two represented the mRNA expression of genes.

### 2.7. SR-BI and LXR*α* Protein Expression Detected by ELISA

The cells in the 6-well plate were sucked into the centrifuge tube, centrifuged at 1 000 r/min at 4°C for 5 min, and the supernatant was discarded. PBS solution was washed 3 times, 100 *μ*L lysate containing PMSF was added to each tube, and the cells were fully contacted by blowing air for 10 seconds (all the above operations were carried out on ice). The 6-well plate was then shaken horizontally to complete cell lysis. After repeated blowing, cell fragments and lysate were moved to a new centrifuge tube as well as centrifuged with 12 000 r/min at 4°C for 5 min. The supernatant was put in a new centrifuge tube and 10 *μ*L was taken for protein determination. The remaining solution was frozen and stored under −70°C for later use. After extracting cytoplasmic proteins, SR-BI and LXR*α* protein expressions were detected based on illustrations of ELISA kit.

### 2.8. Statistics

SPSS 18.0 statistic program was applied for the statistical study of every experimental information. The normality measurement could be conducted on main indicators, one-way ANOVA (*F* test) was used for inter-group contrast, as well as Dunnett-*t* test was applied for multiple contrast. The main data of this experiment were obtained from more than 3 repeated experiments and expressed by mean ± standard deviation.

## 3. Results

### 3.1. Establishment of Macrophage-Derived Foam Cell Model

It could be seen that RAW264.7 macrophages growing along the wall had different cellular morphology, which were mainly round and irregular polygon, and contain 1∼2 nuclei. The cells grew rapidly with prominent pseudopodia and fused in 5∼6 days. After ox-LDL and culture medium were cultured for 48 h, the volume of macrophages increased significantly. and there were lots of lipid droplets in cytoplasm, which could be consistent with morphological characteristics of foam cells. After staining with oil-red O, a large number of red-stained particles appeared in the cells (Figure 1).

### 3.2. Effects of APS on SR-BI and LXR*α*mRNA Expression in Cells

After APS with different concentrations acted on the macrophage origin foam cells for 24 h, expression of SR-BI as well as LXR*α* genes gradually increased with the increase of APS concentration (Figures 2 and 3; Table 1).

### 3.3. Effects of APS on SR-BI and LXR*α* Protein Expression in Foam Cells

With the increase of APS concentration, the protein expressing levels of SR-BI as well as LXR*α* in cells were remarkably higher than those in the control part (*P* < 0.05) (Table 2).

## 4. Discussion

With the improvement of people's living standards and the change in life styles, the morbidity and mortality of cardiovascular diseases are increasing, and AS is the main cause of cardiovascular diseases. The disorder of cholesterol metabolism in macrophages is an important pathogenesis of AS. How to reduce the intake of cholesterol and promote the antitransport of cholesterol is the key to prevent AS [2]. Reverse cholesterol transportation (RCT) refers to procedures in which cholesterol in the extracellular tissues is transferred to the liver through blood circulation and bile acids are produced and discharged out of body, which is the just method for the body to remove excess cholesterol [5].

The effects of SR-BI on the cholesterin antitransport pathway is mainly showed in mediating the outflow of cholesterin from the cells and the selective uptake of cholesterol esters. Research has revealed that the exocellular domain structure of SR-BI exerts a key part in mediating flow of free cholesterol [6], as well as SR-BI could selectively absorb cholesterol through the reverse pinocytosis of HDL [7]. LXR*α* is a component of nuclear hormone acceptor protein family. Studies indicated that LXR is a key receptor and regulatory factor for the body to maintain relatively stable cholesterol, and it can reduce the absorption and utilization of cholesterol, increase the reverse transport, promote the transformation of liver and peripheral tissues, and clear all kinds of low plasma cholesterol levels, thus efficiently inhibiting the formation of lipid plaques and the development of atherosclerosis [4]. Substantial researches have confirmed that activation of LXR can enhance the transcriptional expression of key target genes like ABCAl, ABCGl, ABCG5/G8, apolipoprotein (ApoE), and lipoprotein lipase (LPL). APS is an active ingredient extracted from *Astragalus* membranaceus, and recent studies have found that it exerts an important part in blood lipid regulating as well as the prevention and treatment of AS. APS can inhibit lipid accumulation in macrophages, accelerate cholesterol outflow, and stabilize and decrease the formation of new AS plaques [8, 9]. APS can promote cholesterol efflux from THP-1 macrophages origin foam cells, so it can be speculated that it is associated with the up-regulation of ABCA1 expression [10]. Previous studies have found that APS could reduce the content of cholesterol in foam cells with dose-dependence, as well as the cholesterol efflux promoted by APS may be related to the up-regulation of PPAR*γ* expression [11, 12]. Taking RAW264.7 macrophages as the research object, it showed that contrasted to the control part, APS up-regulated expression of SR-BI and LXR*α* genes and proteins in a dose-dependent manner, consistent with experimental consequences reported in documents. Those outcomes reveal that APS might accelerate cholesterol efflux in macrophages, improve the efficiency of cholesterol antitransportation, and diminish the level of intracellular cholesterol via the up-regulation of the expression of SR-BI and LXR*α*. However, the specific mechanism remains to be further studied.

## Figures and Tables

**Figure 1:** Oil red O staining of RAW264.7 macrophage-derived foam cells (×400).

**Figure 2:** Effects of APS on SR-BI mRNA expression in RAW264.7 macrophages origin foam cells.

**Figure 3:** Effects of APS on LXR*α* mRNA expression in RAW264.7 macrophages origin foam cells.

**Table 1:** The effect of Aps on mRNA expressing levels of SR-BI as well as LXR*α* in RAW264.7 macrophage origin foam cells $\left(\bar{x}\pm s,n=5\right)$

Concentration of APS(mg/L)	SR-BI/*β*-actin	LXR*α*/*β*-actin
0	0.21 ± 0.08	0.25 ± 0.02
10	0.36 ± 0.29^*∗*^	0.34 ± 0.03^*∗*^
20	0.55 + 0.32^*∗*^^#^	0.42 ± 0.03^*∗*^^#^
50	0.82 + 0.51^*∗*^^#△^	0.51 ± 0.05^*∗*^^#△^
100	1.23 + 0.55^*∗*^^#△□^	0.65 ± 0.05^*∗*^^#△□^

^*∗*^ *P* < 0.05, contrast to 0 mg/L; ^#^*P* < 0.05, contrast to 10 mg/L; ^△^*P* < 0.05, contrast to 20 mg/L; ^□^*P* < 0.05, contrast to 50 mg/L.

**Table 2:** The influence of Aps on protein expressing level of SR-BI in RAW264.7 macrophages origin foam cells $\left(\bar{x}\pm s,n=5\right)$

Concentration of APS (mg/L)	Concentration of SR-BI	Concentration of LXR*α*
0	0.5200 ± 0.0171	0.7015 ± 0.0084
10	0.5776 ± 0.0135^*∗*^	0.7336 ± 0.0048^*∗*^
20	0.6129 ± 0.0101^*∗*^^#^	0.7430 ± 0.0013^*∗*^^#^
50	0.6662 ± 0.0114^*∗*^^#△^	0.7517 ± 0.0019^*∗*^^#△^
100	0.7030 ± 0.0222^*∗*^^#△□^	0.7613 ± 0.0028^a^^*∗*^^#△□^

^*∗*^ *P* < 0.05, contrast to 0 mg/L; ^#^*P* < 0.05, contrast to 10 mg/L; ^△^*P* < 0.05, contrast to 20 mg/L; ^□^*P* < 0.05, contrast to 50 mg/L.

## Data Availability

No data are used to support this study.
